The article "Combining Network Pharmacology with Experimental Validation to Elucidate the Mechanism of Salvianolic Acid B in Treating Diabetic Peripheral Neuropathy" was published in 2022. Journal: Evid Based Complement Alternat Med.

# Combining Network Pharmacology with Experimental Validation to Elucidate the Mechanism of Salvianolic Acid B in Treating Diabetic Peripheral Neuropathy

**DOI:** 10.1155/2022/4997327

**Published:** 2022-08-27

**Authors:** Qianqian Wang, Xiaogang Li, Lijun Cao, Yan Li, Yonghui Liu, Lianqing Sun

**Affiliations:** ^1^Department of Traditional Chinese Medicine, The First Affiliated Hospital of Xi'an Jiaotong University, Xi'an 710061, China; ^2^Department of Anesthesiology, The First Affiliated of Xi'an Jiaotong University, Xi'an 710061, China; ^3^Department of Peripheral Vascular, The First Affiliated Hospital of Xi'an Jiaotong University, Xi'an 710061, China

## Abstract

**Background:**

Salvianolic acid B (Sal B) is a bioactive component of Radix Salviae, which has antiinflammation and antiapoptotic activity in diabetic complications. However, the molecular mechanism of action of Sal B on diabetic peripheral neuropathy (DPN) is unknown. This study was designed to identify a mechanism for Sal B in the treatment of DPN by using a pharmacology network, molecular docking, and in vitro experiments.

**Methods:**

Sal B and DPN-related targets from Gene Cards and OMIM platforms were retrieved and screened. Then, an analysis of possible targets with STRING and Cytoscape software was conducted. KEGG signaling pathways were determined using the R software. Subsequently, the binding capacity of Sal B to target proteins was analyzed by molecular docking and in vitro experiments.

**Results:**

A total of 501 targets related to Sal B and 4662 targets related to DPN were identified. Among these targets, 108 intersection targets were shared by Sal B and DPN. After topological and cluster analysis, 11 critical targets were identified, including p38MAPK. KEGG analysis revealed that the AGE-RAGE signaling pathway likely plays an important role in Sal B action on DPN. The p38MAPK protein is a key target in the AGE-RAGE signaling pathway. Molecular docking results suggested that Sal B and p38MAPK have excellent binding affinity (<−5 kcal/mol). The in vitro experiments revealed that Sal B downregulates the expressions of p-P38MAPK, inflammatory cytokines, and apoptosis targets, which are upregulated by hyperglycemia.

**Conclusion:**

Sal B may alter DPN by inhibiting inflammation and apoptosis activated by p38MAPK.

## 1. Introduction

Diabetic peripheral neuropathy (DPN) is the most common microvascular complication in patients with diabetes mellitus (DM), affecting about 50% of cases. It is defined as the emergence of a series of nerve dysfunction in patients with DM. Clinical manifestations include neuropathic pain and sensory disorder or loss. This neuropathic injury greatly affects the patient's quality of life and burdens the family and society. These devastating effects have led to the search for therapeutic solutions [1–3]. Current therapies for DPN include controlled diet, exercise, blood glucose control, and symptomatic drug treatment [4–8]. However, tight glycemic control with insulin increases the risk of severe hypoglycemic episodes and results in treatment-induced neuropathy [9–12]. Further, drug side effects are obvious in intervening in neuropathic pain [13]. Thus, identifying additional drugs that control glucose and have few side effects is needed.

The article "Combining Network Pharmacology with Experimental Validation to Elucidate the Mechanism of Salvianolic Acid B in Treating Diabetic Peripheral Neuropathy" was published in 2022. Journal: Evid Based Complement Alternat Med.

In China, a traditional herb has been widely known and utilized for treating DPN for more than 2000 years because of its prominent efficacy, abundant resources, and low toxicity. Studies showed that traditional herbs lowered patient glucose levels but also relieved the numbness and painful symptoms of DPN [14–16]. Thus, we believe that Traditional Chinese Medicine (TCM) has potential efficacy in the prevention and treatment of DPN. In TCM, DPN belongs to the Xiao-Ke-Bing-Bi-Bing category. Yin fluid deficiency is the main cause of pathogenesis. Yin fluid is a general term for all the normal fluids in the body, which widely exist in all the organs and tissues. Without the cooling influence of yin fluid, the body will become overheated, causing blood coagulation in blood vessels and resulting in ischemic change or neural injury. Thus, promoting blood circulation and clearing coagulated blood are the key treatment points for DPN. Radix Salviae (Danshen in pinyin), the dried root of Salviae Bunge, as shown in Figure 1, is a traditional whole grass herb, presenting satisfactory drug efficacy for curing DPN [17]. Studies showed that Sal B, Salvianolic acid A, Tanshinone IIA, and Tanshinone I were critical components of Radix Salviae, which relieved DM complication symptoms by promoting blood circulation and removing blood coagulation [18]. Salvianolic acid B (Sal B), the chemical structure displayed in Figure 1(b), is the typical bioactive component of Radix Salviae [19]. Modern pharmacology has shown that Sal B contains antiapoptotic, antioxidant, and antiinflammatory properties [20–23]. Previous studies have indicated the effectiveness of Sal B for DM and its complications, especially cardiomyopathy and nephropathy [24, 25]. However, little is known if the antiapoptotic, antioxidant, and antiinflammatory effects are related to the validity of Sal B in treating DPN.

With the rapid progress of bioinformatics and systems biology, a TCM network pharmacology method was created to predict disease-associated genes, detect target profiles of herbal compounds, and elucidate drug-gene-disease comodule associations. This method provides opportunities for discovering bioactive ingredients and biomarkers, potentially revealing scientific evidence of herbal formula-diseases co-action [26]. In this study, we combined computational databases with in vitro experiments to determine the mechanism of Sal B on DPN. We screened the targets of Sal B and DPN by OMIM and Gene Card platforms, collected the critical genes with Cytoscape, and identified possible mechanisms using the Kyoto Encyclopedia of Genes and Genomes (KEGG) analysis. We also validated the predicted results using molecular docking and in vitro experiments. The concrete flow was illustrated in Figure 2. This study provides novel insights into the mechanism of Sal B in the treatment of DPN.

The article "Combining Network Pharmacology with Experimental Validation to Elucidate the Mechanism of Salvianolic Acid B in Treating Diabetic Peripheral Neuropathy" was published in 2022. Journal: Evid Based Complement Alternat Med.

## 2. Materials and Methods

### 2.1. Data Collection and Core Genes Network Construction

To collect the targets of Sal B and DPN, we screened the human gene database (Gene Cards: https://www.genecards.org) and the Online Mendelian Inheritance in Man database (OMIM: https://www.ncbi.nlm.nih.gov/omim). Gene Cards and OMIM databases are considered comprehensive, authoritative compendiums of human genes and genetic phenotypes, which are widely used in analyzing drug components and disease-related targets [27, 28]. “Salvianolic acid B” and “Diabetic peripheral neuropathy” were the keywords. The irrelevant and repeated results were removed manually, and the results were limited to *Homo sapiens*. Then, the intersecting targets between Sal B and DPN were analyzed using a Venn Diagram. After that, the overlapping targets were imported to the String Database (https://string-db.org). The String dataset is one of the largest PPI (protein-protein interactions) datasets, including text mining, experiments, databases, co-expression, neighborhood, gene fusion, and co-occurrence [29]. The scoring condition was designed as >0.40, and selected proteins were limited to “*Homo sapiens*” to ensure the reliability and high confidence of information. All predicted interaction data were uploaded to Cytoscape 3.8.0 software and analyzed by CytoNCA. CytoNCA is a cytoscape plugin for calculation, evaluation, and visualization analysis of multiple centrality measures. Betweenness (BC), Closeness (CC), Degree (DC), Eigenvector (EC), Local Average Connectivity-based method (LAC), and Network (NC) were the major centrality measures. After being evaluated by the above-mentioned standards, the nodes and edges of the data were calculated in the network.

### 2.2. KEGG Pathway Analysis

The mechanisms of action of Sal B on DPN were investigated by using candidate targets transformed to UniProt to collect the target ID codes. Subsequently, the ID codes were analyzed using the R software, which was installed in the Bioconductor database package to get the KEGG signaling pathway. *P* < 0.05 was considered significant.

The article "Combining Network Pharmacology with Experimental Validation to Elucidate the Mechanism of Salvianolic Acid B in Treating Diabetic Peripheral Neuropathy" was published in 2022. Journal: Evid Based Complement Alternat Med.

### 2.3. Component-Target Molecular Docking

The reliability of the predicted interactions between Sal B and p38MAPK was investigated using molecular docking performed with Auto Dock Vina. AutoDock is a molecular docking software that is widely used to predict the binding mode of a ligand in the active site of a protein. The specific procedure is as follows. (1) ligand molecule preparation. The 2D structure of Sal B was explored on the PubChem platform and saved in *∗*sdf format. The 3D structure of Sal B was transformed from the ChemOffice platform and saved in *∗*mol2 format. (2) Receptor molecular preparation. The gene of p38MAPK corresponding protein Q16539 was examined using the UniProt platform. Q16539 corresponding protein 4GEO structure was downloaded in *∗*PDB format. (3) Molecular docking. The PDB format of the receptor with added polar hydrogen, removed solvent, and organics were saved as the receptor PDBQT format. Then, the mol2 format was transformed to the ligand PDBQT format similarly. Next, the ligand PDBQT-receptor PDBQT format docking box was constructed in Auto Grid, and the docking results were displayed in PYMOL software.

### 2.4. Cell Culture and Drug Treatment

RSC96 cells were purchased from Shan-Xi-Fan-Chang-Sheng-Wu and cultivated in DMEM medium (Life Technologies, USA) with 10% fetal calf serum (Life Technologies, USA) at 37°C in an atmosphere comprising 5% CO_2_. Cells were cultured with different solutions, and the groups were arranged as follows: control (5.6 mmol/L glucose), high glucose (HG, 125 mmol/L glucose), and Sal B (125 mmol/L glucose with 1 *μ*mol/L Sal B (Aladdin, China)).

### 2.5. Immunofluorescence Analysis

Cells were cultured at a 5.0 × 10^5^ density in 9.6 cm dishes. After the cells were completely adhered to the wall, the cells were treated with different solutions as the above-mentioned. Then, the cells were incubated with primary antibodies (1 : 200, Caspase 3, affinity, USA) and secondary antibodies (1 : 250, Abways, China). The nuclei were stained with 4′,6-diamidino-2-phenylindole (DAPI) (Servicebio, China). After that, the cells were fixed with an embedding medium on a microscope slide and imaged by fluorescent microscopy (Nikon Corporation, Japan).

### 2.6. Enzyme-Linked Immunosorbent Assay (ELISA)

The cells were cultured at a 5.0 × 10^5^ density in 9.6 cm dishes and incubated for analysis. The levels of IL-6 and IL-1*β* in cell supernatants were extracted and quantified with commercial ELISA kits (Enzyme-Linked Biotechnology, Shanghai, China), following the manufacturer's protocol.

The article "Combining Network Pharmacology with Experimental Validation to Elucidate the Mechanism of Salvianolic Acid B in Treating Diabetic Peripheral Neuropathy" was published in 2022. Journal: Evid Based Complement Alternat Med.

### 2.7. Western Blot Analysis

The cells were cultured at a 5.0 × 10^5^ density in 9.6 cm dishes and then lysed and extracted. The BCA assay was used to quantify proteins. Proteins were loaded on an SDS-PAGE polyacrylamide gel, transferred to an NC membrane (Pall Corporation, USA), incubated with p-P38MAPK (1 : 1000) antibodies, and subsequently measured by chemiluminescence (ECL, Sheng-Er-biology, China). Images were analyzed by Image-Lab software (Bio-Rad, Hercules, CA, USA).

### 2.8. Statistical Analysis

All values were exhibited as mean ± SD. Experiments were repeated at least three times. Data were analyzed by SPSS 18.0, and differences among groups were analyzed by one-way analysis of variance (ANOVA). Statistical analyses were performed using the GraphPad 5 software, with *P* < 0.05 being considered statistically significant (see Figures1 and 2).

## 3. Results

### 3.1. Identification of Targets of DPN and Sal B in Various Databases

In total, we discovered 501 potential targets of Sal B after removing duplicate data. There were 453 targets in OMIM and 51 in Gene Cards. A total of 4662 targets related to DPN were identified after removing duplicate data. There were 409 targets in OMIM and 4352 in Gene Cards. Comparison of the 501 potential targets of Sal B with the 4662 identified with DPN resulted in 108 overlapping targets detected by Venn Diagram (Figure 3).

### 3.2. Establishment of the Critical Targets Network of Sal B Action on DPN

The overlapping targets between Sal B and DPN were uploaded to the STRING platform. The interaction files were imported to Cytoscape software. When the criteria were set at Betweenness (BC): 28.003, Closeness (CC): 0.4049, Degree (DC): 6, Eigenvector (EC): 0.03229, Local Average Connectivity-based method (LAC): 2.125, and Network (NC): 3, the results presented in Figure 4(a), indicate 100 nodes and 512 edges. When the screening criteria were set at Betweenness (BC): 6.268, Closeness (CC): 0.673, Degree (DC): 17, Eigenvector (EC): 0.1727, Local Average Connectivity-based method (LAC): 12.8, and Network (NC): 14.445, the results shown in Figure 4(b) indicated 34 nodes and 286 edges. After screening by the above procedure, the ultimate critical targets are presented in Figure 4(c).

### 3.3. KEGG Classification of Target Proteins

To further identify a mechanism of action for Sal B on DPN, the ID codes between Sal B and DPN were uploaded to R software, and the top 20 signaling pathways were determined (Figure 5(a)). Among the pathways, the AGE-RAGE signaling one in diabetic complications was critical, as presented in Figure 5(b).

The article "Combining Network Pharmacology with Experimental Validation to Elucidate the Mechanism of Salvianolic Acid B in Treating Diabetic Peripheral Neuropathy" was published in 2022. Journal: Evid Based Complement Alternat Med.

### 3.4. Molecular Docking of Sal B Action on the p38MAPK Protein

Molecular docking of Sal B action on p38MAPK was generated with Auto Dock software. The binding energy values of Sal B and p38MAPK (−9.1 kcal/mol) showed that the former interacts with the p38MAPK receptor. The 2D structure of Sal B was downloaded from the PubChem platform and the 3D structure was transformed in ChemOffice (Figure 6(a)). The p38MAPK protein was also downloaded on the PDB platform. After adding polar hydrogen and removing solvent and organic in PYMOL software, p38MAPK protein was constructed (Figure 6(b)). The binding box of Sal B and p38MAPK was constructed in Auto Dock software. The binding box-related files were analyzed in Auto Dock Vina, and a PDBQT file was generated (Table 1). Next, the receptor and ligand PDBPT files were analyzed in PYMOL software (Figure 6(c)).

### 3.5. Validation of the Potential Mechanism of Sal B Action on DPN

Combining critical targets and signaling pathway results indicated p38MAPK, Caspase 3, IL-6, and IL-1*β* as targets and verified by in vitro analysis. The level of p-p38MAPK was determined by western blot. Results showed that p-p38MAPK was low in control cells but increased in hyperglycemic conditions. The addition of Sal B lowered the expression of p-P38MAPK, as shown in Figure 5(a). Proteins downstream of p-P38MAPK, including caspase 3, IL-6, and IL-1*β*, were analyzed by immunofluorescence and ELISA. Results showed that caspase-3, IL-6, and IL-1*β* were low in controls but increased in hyperglycemic conditions. Again, the addition of Sal B lowered the levels of caspase-3, IL-6, and IL-1*β* as shown in Figures 7(b)–7(d).

## 4. Discussion

DPN is the most common complication of DM. Although many studies using in vitro and in vivo models have been done, there is no effective treatment for DPN. Sal B, the main component of Radix Salviae, has been identified as being neuroprotective both in vitro and in vivo [30]. However, there is little information regarding the neuroprotective effects of Sal B in high glucose-treated Schwann cells (SCs). Our data shows that the protective effects of Sal B on DPN are associated with apoptosis and the inflammatory processes, which are regulated by p38MAPK.

Studies have shown that the p38MAPK receptor initiates inflammatory cytokine (IL-6, IL-1*β*, and TNF-*α*) released in diabetic complications [31, 32]. Our pharmacology network results showed that inflammatory cytokine released by induction of p38MAPK is a critical process in Sal B signaling in DPN. To validate this result, SCs were used to imitate a DPN model. SCs are sensitive to glucose concentration as studies revealed that 30–150 mM glucose concentrations are suitable for inducing DPN [33–39]. Our previous studies indicated a concentration of hyperglycemia in SCs that resulted in detrimental effects at 125 mmol/L glucose for 72 h. Thus, 125 mmol/L glucose was considered an appropriate concentration that resulted in neuronal injury. The results here showed that the levels of p38MAPK, IL-6, and IL-1*β* were upregulated after treatment with high glucose. Addition of Sal B results in both p38MAPK and inflammatory cytokines being significantly downregulated compared with untreated SCs. Studies also revealed that the release of apoptosis mediators driven by the phosphorylation of p38MAPK induced neuropathy [40, 41]. In our experiments, immunofluorescence assays showed that the expression of caspase-3 in hyperglycemic conditions is significantly increased. After treatment with Sal B, the expression of caspase-3 was reduced. These results indicate that p38MAPK is the critical bridge between the regulation of inflammation and apoptosis in DPN. The mechanism of action of Sal B on DPN is related to p38MAPK targets. Binding positions between Sal B and p38MAPK were analyzed by molecular docking. A negative interaction energy (−9.1 kcal/mol) for the docked-complexes calculated with AutoDock indicated an efficient interaction between Sal B and p38MAPK.

The article "Combining Network Pharmacology with Experimental Validation to Elucidate the Mechanism of Salvianolic Acid B in Treating Diabetic Peripheral Neuropathy" was published in 2022. Journal: Evid Based Complement Alternat Med.

The inhibition of inflammation, apoptosis, and phosphorylation of p38MAPK by Sal B has been studied previously [22, 42–45]. However, it has not been analyzed by combining a computation database with experimental validation. The network pharmacology evaluation method guidance indicates that the reliability and repeatability should be mainly evaluated by model construction. The evaluation model includes computer model construction, in vitro and in vivo experiments, and a clinical research cohort. In this study, we adopted the pharmacology network, molecular docking, and in vitro experiments together, and concluded that Sal B might limit DPN by inhibiting inflammation and apoptosis through p38MAPK. Although we examined the predicted results of Sal B in an SC model, no experiments in which Sal B was used on animals or humans were performed. This study does suggest that hyperglycemia activates inflammation and apoptosis through the p38MAPK pathway. Future studies will need to address these limitations and investigate the mechanism of Sal B acting on DPN in vivo.

In summary, Sal B treatment decreased the upregulation of the p38MAPK receptor in SCs and decreased its mediated inflammation and apoptosis activation. These results provide a theoretical basis for Sal B research and its clinical application in DPN.

## 5. Conclusion

In conclusion, the pharmacology network, molecular docking, and in vitro experimental analysis identify potential molecular mechanisms of Sal B in the treatment of DPN. Sal B may limit inflammation and apoptosis by adjusting p38MAPK. This provides a theoretical basis for the ameliorative effect of Sal B on DPN.

The article "Combining Network Pharmacology with Experimental Validation to Elucidate the Mechanism of Salvianolic Acid B in Treating Diabetic Peripheral Neuropathy" was published in 2022. Journal: Evid Based Complement Alternat Med.

## Figures and Tables

**Figure 1:** The natural origin and chemical structure of Sal B. (a) A picture of *Salvia miltiorrhiza*; (b) the chemical structure of Sal B.

**Figure 2:** The whole framework of this study is based on the methods of network pharmacology, molecular docking, and experimental verification.

**Figure 3:** Venn diagram analysis results. The blue color represents Sal B-related targets, the pink color represents the DPN-related targets, and the middle red color represents the overlapping targets between Sal B and DPN.

**Figure 4:** The gene mutual network result. The lines between genes represent the edges. The genes in the boxes represent the nodes. Among these boxes, the yellow boxes represent the critical genes screened by betweenness (BC), closeness (CC), degree (DC), eigenvector (EC), local average connectivity-based method (LAC), and network (NC). The screened targets were the critical targets in Sal B acting on DPN.

**Figure 5:** (a) The bubble chart of the top 20 KEGG pathways. The circle size represents the critical size of the KEGG pathway. (b) The critical genes of the AGE-RAGE signaling pathway in diabetic complications. The red square genes represent the critical genes which are involved in the AGE-RAGE signaling pathway in diabetic complications.

**Figure 6:** Molecular docking of Sal B on P38MAPK corresponding protein. A simulated model of Sal B docked with the P38MAPK protein generated using a computer. (a) The 3D structure of Sal B; (b) the structure of P38MAPK corresponding protein; and (c) the best docking position for Sal B on the P38MAPK protein. The results showed that Sal B could interact with the P38MAPK protein.

**Figure 7:** (a) Western blot for the expression of p-P38MAPK in RSC96 cells. (^*∗*^*P* < 0.05, compared with the control group; ^#^*P* < 0.05, compared with the HG group). Values are mean ± SD, *n* = 3. (b) The immunofluorescence analysis of caspase-3. The red color represents caspase-3 and the blue color represents DAPI. Merge is the overlapping of the red and blue colors. (c, d) ELISA analysis of IL-6 and IL-1*β* in RSC96 cells. (^*∗*^*P* < 0.05, compared with the control group; ^#^*P* < 0.05, compared with the HG group). Values are mean ± SD, *n* = 3.

**Table 1:** MOE score of P38MAPK protein and Sal B (kcal/mol).

Mode	Affinity (Kcal/mol)	Dist from best mode	
		RMSD l. b.	RMSD u. b.
1	−9.1	0.00	0.00
2	−8.8	1.829	3.552
3	−8.7	1.284	2.198
4	−8.6	12.786	16.269
5	−8.5	12.788	17.037
6	−8.2	12.361	15.144
7	−8.2	2.494	3.720
8	−8.1	1.974	4.141
9	−8.0	12.552	17.086
10	−8.0	12.220	17.083
11	−7.9	13.182	17.421
12	−7.9	3.612	8.240
13	−7.8	17.813	21.386
14	−7.8	2.868	10.412
15	−7.7	11.648	17.590
16	−7.7	18.389	23.051
17	−7.7	3.125	8.132
18	−7.7	3.829	7.618
19	−7.7	5.374	9.620
20	−7.5	5.030	9.639

*Note*. The predicted binding affinity is in kcal/mol (energy). RMSD values are calculated relative to the best mode and use only movable heavy atoms. Two variants of RMSD metrics are provided, RMSD/l. b. (RMSD lower bound) and RMSD/u. b. (RMSD upper bound), differing in how the atoms are matched in the distance calculation. RMSD: root-mean-square deviation.

The article "Combining Network Pharmacology with Experimental Validation to Elucidate the Mechanism of Salvianolic Acid B in Treating Diabetic Peripheral Neuropathy" was published in 2022. Journal: Evid Based Complement Alternat Med.

## Data Availability

The data used to support the findings of this study are open. The links to the databases are available at the corresponding locations in the original text.
